RETRACTED

# Clinical Characteristics and Drug Resistance Analysis of 90 Cases of Children with Salmonella Enteritis

**DOI:** 10.1155/2022/5091945

**Published:** 2022-08-03

**Authors:** Yang Wang, Wei Zhang

**Affiliations:** ^1^Maternal and Child Health Hospital of Hubei Province, China; ^2^Women and Children's Hospital of Hubei Province, China; ^3^Tongji Medical College, Huazhong University of Science and Technology, China

## Abstract

**Objective:**

To summarize the clinical characteristics and drug sensitivity analysis of children with Salmonella enteritis in our hospital, explore the characteristics and drug resistance of Salmonella infection, and guide the rational clinical use of drugs.

**Methods:**

The clinical data of 90 pediatric Salmonella enteritis patients treated in our hospital from January 2015 to January 2020 were selected as the observation group of this retrospective study, and 90 patients with non-Salmonella enteritis were selected at the same time as a control group. Discuss the clinical characteristics of Salmonella, drug sensitivity analysis, infection characteristics, and drug resistance and guide the rational clinical use of drugs.

**Results:**

The susceptibility rates of 15 antibiotics from high to low were imipenem and meropenem, piperacillin, cefoperazone, compound trimethoprim, chloramphenicol, and ceftazidime. Salmonella strains were both resistant to imipenem and meropenem. Salmonella is sensitive and has a low rate of resistance to quinolones (ciprofloxacin) and a high rate of resistance to cephalosporins (ceftriaxone, cefotaxime, ceftazime, and cefpiramide), both reached more than 28%. Salmonella has the highest resistance to penicillin and erythromycin, both at 85.00% and above. Among 90 children with Salmonella enteritidis food poisoning, 32 were hospitalized, 21 cases were hospitalized less than 7 days, and 11 cases were 7-14 days. The longest hospital stay was 12 days, the shortest was 1 day, and the average was 6.1 days. Seven people stayed for observation and 51 people were discharged after treatment. All the children recovered without death.

**Conclusion:**

In clinical practice, antibiotics should be used rationally based on drug susceptibility results. In the case of poor efficacy of cephalosporins, amoxicillin and potassium clavulanate, piperacillin, tazobactam, or imipenem, cephalosporin antibiotics can be considered the first choice for clinical empiric medication.

## 1. Introduction

Salmonella is an intestinal pathogen with a wide distribution, multiple serotypes, and complex antigens. It can cause human gastroenteritis, bloodstream infections, and food poisoning. It is one of the most common pathogens of food-borne diarrhea globally [1]. Salmonella is a common disease and frequently occurring disease in my country and worldwide. More than 1/3 of Salmonella infections occur in children under 10 years old, and the infection rate of infants under 1 year old is more than 10 times higher than that of the general population [2]. Because the bacteria have a wide range of hosts, it is currently the most isolated type of bacteria in various countries, and the bacteria are highly adaptable and tolerant to the external environment. Compared with other bacterial enteritis, this type of bacteria infection diarrhea lasts for a long time, it is not easy to get good control, and it will not heal [3]. Salmonella is easy to spread through food to cause digestive tract infections, and infants and young children with imperfect immune function development are susceptible to Salmonella [4]. In recent years, the overuse and abuse of antibacterial drugs have led to the continuous increase of drug resistance of Salmonella and even the emergence of multidrug-resistant bacteria including fluoroquinolones and cephalosporins, which has brought certain difficulties to the clinical treatment of patients [5]. In recent years, the incidence of Salmonella enteritis has shown an obvious upward trend [6]. Different from other studies, this study examined Salmonella patients, analyzed the clinical characteristics and infection characteristics of Salmonella, and then guided the rational clinical use of drugs by analyzing their susceptibility and drug resistance, further rationalizing the use of antibiotics and avoiding the possibility of wrong treatment. Based on this, our hospital is aimed at investigating the clinical characteristics of children with Salmonella enteritis in our hospital and analysis of drug susceptibility, exploring the characteristics of Salmonella infection and drug resistance, and guiding the rational clinical use of drugs. The current research results are reported as follows.

RETRACTED

## 2. Materials and Methods

### 2.1. General Information

We review the hospitalized medical records of patient 1 and collect and analyze the clinical data of patient 1 with confirmed Salmonella enteritis, including age, gender, personal history, medical history, clinical symptoms, signs, and auxiliary examination and treatment information. Ninety Salmonella enteritidis food poisoning cases were all outpatient and emergency outpatients in this hospital. Fifty-three boys (58.9%) and 37 girls (41.1%). Eight cases (8.9%) aged 2 to 3 years old (elementary class), 37 cases (41.1%) aged 3 to 4 years old (small class), 23 cases (25.6%) aged 4 to 5 years (medium class), and 22 cases (24.4%) aged 5-6 years old (large class) (Table 1). Bacterial culture and identification are performed by the third edition of the “National Clinical Laboratory Procedures” for standard operations [7]. The Microscan96 automatic bacterial susceptibility test was used for the susceptibility test, and the results were judged according to the standards of the Clinical Laboratory Standards Institute (CLSI) (2012) [8]. All patients were asked about their medical history and physical examination in detail, and relevant records were made.

### 2.2. Sources of Strains and Reagents

The clinical data of 90 pediatric Salmonella enteritis patients treated in our hospital from January 2015 to January 2020 were selected, and the previously detected cases were collected for statistical analysis. Reagents and equipment are as follows: medium xylose-lysine-deoxycholic acid agar (XLD), Salmonella chromogenic medium, MH agar and modified selenite yellow-green enrichment broth (SBG), Salmonella biochemical identification kit (Guangdong Huankai Microbial Technology Co., Ltd.), drug-sensitive paper (Oxoid, UK), and Salmonella diagnostic serum (Ningbo Tianrun Biopharmaceutical Co., Ltd.); quality control strain is Escherichia coli ATCC25922 (purchased from Guangdong Clinical Laboratory Center); VITEK automatic bacterial identification instrument (Merieux, France) and Microscan automatic bacterial identification instrument (Siemens, USA) were also used.

### 2.3. Method

Separation culture and serological typing: pick the stool with pus, blood, or mucus, take the liquid stool and flocculate in a sterile container, and send it for inspection in time; if you use a rectal swab, you need to clean the anus with soapy water and use it to increase bacteria. The liquid-moistened anal sampling swab is inserted into the anus 2 ~ 3 cm, gently rotated, and placed in the Cary-Blair transport medium. Then, inoculate the XLD plate and SBG enrichment solution for culture. Take the suspicious colony on the XLD plate (the black transparent in the center, smooth, moist, neat edge, round colony) or SBG incubate for 16~18 h to increase the bacteria, then streak and inoculate to the Salmonella chromogenic plate. Take the suspicious colony on the chromogenic plate (2 ~ 3 mm purple-red colony), use the Salmonella biochemical identification kit for preliminary identification, select the suspicious Salmonella with a red slope on the trisaccharide iron agar, yellow bottom with gas production, and hydrogen sulfide positive, and use the automatic bacterial identification instrument to identify the suspected Salmonella. After Salmonella, use Salmonella diagnostic serum for typing (some strains require continuous induction to determine the flagella phase 2). According to the White-Kauffmann-Le-Minor (WKLM) antigen table, the serotype of each strain of Salmonella was determined. For drug susceptibility test, the Kirby-Bauer method recommended by WHO was used for the Salmonella susceptibility test, and the results were judged based on the American Society for Clinical Laboratory Standardization (CLSI 2012 edition). The quality control strain is Escherichia coli ATCC25922.

RETRACTED

### 2.4. Observation Indicators

In pathogen detection, collect the patient's stool and send it for inspection immediately. The detection of pathogenic bacteria is mainly an automatic bacteria analyzer for drug susceptibility testing, and the agar disc diffusion method is mainly used for detection. Three consecutive inoculations were made on blood, blue, and chocolate plates. They were separated after incubating at 35°C for 1 day and were identified by traditional methods. The suspicious strains were identified through Gram staining and biochemical reaction, and the same strain was determined to be the pathogenic strain in two consecutive tests.

### 2.5. Statistical Methods

The data in this study was calculated using Excel and reviewed by two physicians. The selected data follow the normal distribution. After the first author and corresponding author have entered the data into the computer system and proofread, the statistical software is used for SPSS25.0 to perform related calculations. The measurement data were expressed as mean ± standard deviation ($\bar{x}\pm S$) by independent sample *t*-test, and count data expressed as a percentage (%) or integer were used by *χ*^2^ test. Statistical *P* < 0.05 indicated that the difference was statistically significant.

## 3. Results

### 3.1. Clinical Characteristics of Salmonella

Among the 90 children with Salmonella enteritis, the youngest onset was 7 months and the oldest was 4 years and 11 months; children under 2 years old were the main patients. Diarrhea occurred in the 90 cases, and the stool characteristics and colors were changeable, which could be watery stools, yellow egg-patterned stools, yellow-green mucus stools, mucous pus and bloody stools, or bloody stools. Among them, 83 children had mucous pus and bloody stools. 69 children had a fever, of which 61 children had a fever above 39°C, and the fever lasted 3 to 5 days after treatment. Other symptoms include vomiting, abdominal pain, abdominal distension, dehydration, and convulsions and those with respiratory infections. All children were instilled with antibiotics to fight infections (mainly third-generation cephalosporins), and 7 cases were completely resistant to third-generation cephalosporins. Some children with resistant strains had repeated illnesses and prolonged courses of disease. According to the drug sensitivity test results, the clinical symptoms were finally relieved after switching to meropenem and other treatments. The median hospitalization time was 8 days (4-16 days), and the median time of stool formation was 8 days (3-14 days). Ninety children with stool formation and general recovery were discharged after negative reexaminations of double fecal cultures.

RETRACTED

### 3.2. Antibiotic Resistance Rate of Salmonella

The susceptibility rates of 15 antibiotics from high to low are imipenem and meropenem, piperacillin, cefoperazone, compound trimethoprim, chloramphenicol, and ceftazidime. Salmonella strains are sensitive to both imipenem and meropenem. The drug resistance rate to ampicillin and piperacillin is relatively high. Only 2 strains are sensitive to all tested antibiotics. One strain was resistant to 9 antimicrobials and was only susceptible to piperacillin/tazobactam, imipenem, and meropenem. Salmonella has a low resistance rate to quinolones (ciprofloxacin) and a high resistance rate to cephalosporins. The resistance rates to ceftriaxone, cefotaxime, ceftazidime, and cefepime are all up to more than 28%, see Figure 1.

### 3.3. Analysis of Salmonella Resistance

Salmonella has the highest resistance to penicillin and erythromycin, both at 85.00% and above, see Figure 2.

### 3.4. Clinical Efficacy

Among 90 children with Salmonella enteritidis food poisoning, 32 were hospitalized, 21 cases were hospitalized for less than 7 days, and 11 cases were 7-14 days. The longest hospital stay was 12 days, the shortest was 1 day, and the average was 6.1 days. Seven people stayed for observation, and 51 people were discharged after treatment. All the children recovered without death (Table 2).

### 3.5. Case Analysis

Patient Gao, female, 5 years old, was given “Merrill Lynch” because of “intermittent fever for 4 days and abdominal pain for 3 days.” The child developed fever 4 days ago without an obvious cause, with a maximum body temperature of 39.0°C, accompanied by cold limbs and no convulsions. After treatment, “antipyretic suppository” can be reduced to normal, easy to repeat, accompanied by vomiting once, a small amount of stomach content, no bile and coffee grounds, and a yellow paste-like stool, no mucus and bloodshot eyes, no abdominal pain, no cough, expectoration, no nasal congestion, and runny nose. Later, I took medicine “Honeysuckle Oral Liquid, Jianwei Granules” twice in the outpatient department of Hubei Provincial Hospital of Traditional Chinese Medicine. No obvious improvement was observed. Abdominal pain occurred 3 days ago, mainly around the umbilical cord. It is irrelevant. I relieved 2 times of yellow watery stool without mucus or blood streaks. Later, in our hospital outpatient clinic, he was treated with “Utanen and Oxican” infusion treatment for 2 days (May 16-17). I vomited 2 times after drinking water yesterday. It is a small number of stomach contents. During the pharyngeal examination, a small number of stomach contents was vomited. The child still has a fever and no vomiting. Today, he relieved a small amount of yellow mushy stool and still complained of abdominal pain. The degree of abdominal pain and the frequency of abdominal pain are relatively high. Exacerbation, preliminary diagnosis: (1) acute gastroenteritis, acute mesenteric lymphadenitis. She was admitted to the hospital with “intermittent fever for 4 days and abdominal pain for 3 days.” Admission examination: *T* 36.3°C, P126 beats/min, R22 beats/min, clear, good reaction, no dehydration, no skin rash on the whole body, no enlarged lymph nodes on the neck, soft neck, no chapped lips, no Bayberry tongue, pharyngeal hyperemia, swollen tonsils, no purulent secretions, thick breath sounds in both lungs, no rales, strong heart sounds, heart rate 126 beats/min, regular rhythm, no pathological murmurs, and a flat abdomen. The muscles are slightly tense and tender, with obvious tenderness around the umbilical cord, Mack's point tenderness (±), rebound pain (-), and normal bowel sounds. The extremities can circulate in the extremities, and the pathological signs are not elicited. There is no hard swelling on the fingertips and no molting around the anus. After admission, anti-infective treatment was performed with cefoperazone and tazobactam sodium and symptomatic and supportive treatment with fluid rehydration. The child had no symptoms such as fever, abdominal pain, or diarrhea. The general condition is okay. Reexamining stool culture did not detect Salmonella, which reached the clinic healed and was discharged.

RETRACTED

## 4. Discussion

Salmonella is one of the main pathogens of bacterial enteritis in children. Salmonella is widespread in nature. In addition to infecting humans, it can also infect many animals. If you eat meat, eggs, dairy products, and other foods contaminated with Salmonella, later, it can cause infection. Most Salmonella infections are related to an unclean diet, so it is particularly important to control the source of infection, prevent food contamination, and cut off the transmission route of bacteria [9].

Among the 90 children with Salmonella enteritis in this study, the youngest onset was 7 months and the oldest was 4 years and 11 months; children under 2 years old were the main patients. The children had diarrhea during the disease, and the stool characteristics and colors were changeable, which could be watery stools, yellow egg-patterned stools, yellow-green mucus stools, mucus pus and bloody stools, or bloody stools. Among them, 83 children had mucus pus and bloody stools. 69 children had a fever, of which 61 children had a high fever above 39°C. After treatment, the high fever lasted for 3 to 5 days. Other symptoms included vomiting, abdominal pain, abdominal distension, dehydration, convulsions, and respiratory infections. The cases in this study had a rapid onset and rapid progress, with an incubation period of 2.5 to 32 hours, with fever at the beginning of the disease, and most of them showed persistent high fever. Diarrhea is mostly watery yellow stools and sloppy stools, some mucus stools or bloodshot mucus stools, with or without abdominal pain and vomiting, a small number of patients have skin rashes, and the course of the disease is 1 to 2 weeks [10]. Salmonella enteritidis food poisoning mainly manifests as digestive tract symptoms and fever. Pathogenic bacteria multiply in the human intestine and release endotoxins that can cause diarrhea, abdominal pain, vomiting, and other digestive system symptoms, which have a strong stimulating effect on the intestinal mucosa, intestinal wall nerves, and blood vessels, causing swelling and exudation of the intestinal mucosa, as well as dysfunction [11]. At the same time, endotoxin is absorbed into the blood from the intestinal wall and acts on the body temperature regulation center and vascular motor nerves through circulation, causing symptoms such as fever and dehydration [12].

The susceptibility rates of the 15 antibiotics in this study from high to low were imipenem and meropenem, piperacillin, cefoperazone, compound trimethoprim, chloramphenicol, and ceftazidime. Salmonella strains were both resistant to imipenem and meropenem. Sensitive, high resistance rate to ampicillin and piperacillin, only 2 strains are sensitive to all tested antibiotics, of which 1 strain is resistant to 9 kinds of antibacterial drugs, and only to piperacillin, imipenem, and meropenem is sensitive. The less use of azithromycin in treating Salmonella infections is related to the high sensitivity rate, suggesting that azithromycin can be added in the drug susceptibility test. In terms of treatment, according to the results of drug susceptibility, azithromycin can be used for anti-infection treatment if necessary. Of course, the difference in antimicrobial resistance rates mentioned in the study is related to the identification methods and evaluation criteria used in the drug susceptibility test. However, these data are of great significance for the guidance of clinical empirical treatment and the selection of antimicrobial drugs [13]. Therefore, focusing on continuous monitoring of Salmonella infection and drug resistance, targeted selection of antibacterial drugs, and understanding of the resistance of bacteria in the region will provide clinicians with strong guidance on drug use, which can promptly and effectively treat and prevent serious diseases. The occurrence of complications [14]. Salmonella infections have been increasing year by year in Xi'an in recent years. The characteristics and color of the stools in children are changeable. The stool is mostly pus and blood. It is not easy to distinguish from bacillary dysentery. At the same time, it is accompanied by high heat peaks, a long course of the disease, difficult to control and unhealed condition, but rarely affects important organs such as the liver and heart. Multiple drug-resistant strains are increasing year by year [15]. The resistance of the third-generation cephalosporins, which are currently used mainly in children, poses challenges for clinicians. Strengthening the monitoring of bacterial resistance and epidemiological investigations, early diagnosis, reasonable full course of treatment, and selection of sensitive antibiotics to fight infection are the keys to controlling Salmonella infection [16].

RETRACTED

There are also some shortcomings in the study, antibacterial treatment is not a conventional means of Salmonella gastroenteritis, antibacterial intervention may prolong the excretion of bacteria from the intestine, but if an invasive infection requires the immediate use of antibacterial drugs, whether the results of this study are still suitable for guiding clinical medication is still unclear. Therefore, different symptoms should also be further studied. There are many different types of Salmonella, and their infectivity is also different, so there are great differences in the choice of medication, and similarly, the age of children also has a great influence on the choice of medication, which are the problems to be considered in guiding the use of Salmonella in children.

To sum up, the incidence of Salmonella enteritis is increasing year by year. Children under 2 years old are susceptible to Salmonella infection, stool characteristics and color are changeable, the disease course is long, and the multidrug-resistant strains increase year by year. It is difficult to control and the disease is prone to prolong and unhealed. Clinicians should choose sensitive antibiotics rationally and cautiously based on the results of drug susceptibility tests. They should use antibiotics reasonably based on drug susceptibility results in clinical practice. Cephalosporin antibiotics can be used as the first choice for clinical experience medication. In the case of poor efficacy of cephalosporin, amoxicillin, and clavulanate potassium, piperacillin, tazobactam, or imipenem can be considered.

RETRACTED

## Figures and Tables

**Figure 1:** Antibiotic resistance rate of Salmonella.

**Figure 2:** Comparison of drug resistance of Salmonella (%).

**Table 1:** Basic information on 90 cases of Salmonella enteritidis food poisoning.

Age	Grade	Case	Percentage (%)
2-3 years old	Elementary class	8	8.9%
3-4 years old	Small class	37	41.1%
4-5 years old	Medium class	23	25.6%
5-6 years old	Large class	22	24.4%

**Table 2:** Treatment of 90 children with Salmonella enteritidis food poisoning.

Treatment situation	Case
Hospitalization less than 7 days	21
Hospitalization for 7-14 days	11
Discharged after treatment	7
Stayed for observation	51

## Data Availability

The datasets used and analyzed during the current study are available from the corresponding author upon reasonable request.
